The article "Design, Synthesis, and Biological Evaluation of (E)-N'-((1-Chloro-3,4-Dihydronaphthalen-2-yl)Methylene)Benzohydrazide Derivatives as Anti-prostate Cancer Agents" was retracted in 2023. Reasons: original data or images not available; unreliable data; unreliable results or conclusions; concerns about the images.

# Design, Synthesis, and Biological Evaluation of (E)-N'-((1-Chloro-3,4-Dihydronaphthalen-2-yl)Methylene)Benzohydrazide Derivatives as Anti-prostate Cancer Agents

**DOI:** 10.3389/fchem.2019.00474

**Published:** 2019-07-10

**Authors:** H. A. Arjun, Ramakrishnan Elancheran, N. Manikandan, K. Lakshmithendral, Muthiah Ramanathan, Atanu Bhattacharjee, N. K. Lokanath, Senthamaraikannan Kabilan

**Affiliations:** ^1^Drug Discovery Lab, Department of Chemistry, Annamalai University, Chidambaram, India; ^2^Department of Pharmacology, PSG College of Pharmacy, Coimbatore, India; ^3^Computational Biology Laboratory, Department of Biotechnology & Bioinformatics, North Eastern Hill University, Shillong, India; ^4^Department of Physics, University of Mysore, Mysore, India

**Keywords:** androgen receptor, prostate cancer, benzohydrazide, molecular docking, molecular dynamics, ADME

## Abstract

Prostate Cancer (PCa) is the most frequently diagnosed cancer in men in their late '50s. PCa growth is mainly due to the activation of the androgen receptor by androgens. The treatment for PCa may involve surgery, hormonal therapy, and oral chemotherapeutic drugs. A structural based molecular docking approach revealed the findings of *(E)-N'-((1-chloro-3,4-dihydronaphthalen-2-yl)methylene)benzohydrazide* derivatives, where the possible binding modes of the compounds with protein (PDB ID: 3V49) are shown. The compounds (*6a-k*) were synthesized and characterized by using conventional methods. The compounds, *6g, 6j*, and *6k* were reconfirmed through single crystal X-ray diffraction (XRD). Further, the compounds *(6a-k)* and standard drug were evaluated against human prostate cancer cell lines, LNCaP and PC-3 and the non-cancerous cell line, 3T3. Among these compounds, *6g* and *6j* showed higher cytotoxicity, and *6g* exhibited dose-dependent activity and reduced cell viability. The mechanism of action was observed through the induced apoptosis and was further confirmed by western blot and ELISA. Molecular dynamics simulation studies were carried out to calculate the interaction and the stability of the protein-ligand complex in motion. ADME properties were predicted for all the tested compounds. These findings may give vital information for further development.

## Introduction

Cancer is a group of heterogeneous diseases leading to abnormal cell growth and dysfunction which proliferates to other parts of the body. Prostate cancer (PCa) is the second leading cause of cancer deaths among men in the United States. The American Cancer Society has estimated that 174,650 men will be diagnosed and there will be 31,620 deaths due to PCa in the United States in 2019 (American Cancer Society, 2019). Androgens, Dihydrotestosterone (DHT), and testosterone bind with the ligand binding domain of the androgen receptor (AR) and stimulate the growth of prostate cancer (Ferlay et al., 2010; Elancheran et al., 2015). The AR agonist and antagonist bind to the same binding pocket, but the AR antagonist is made of bulkier molecules than the AR agonist. Therefore, the AR agonist prevents the closing of helix-12 toward the ligand binding domain (Bohl et al., 2005). Thus, AR antagonists such as bicalutamide, enzalutamide, and flutamide prevent the activation of the androgen receptor. The mutation at amino acids Threonine 877 and Tryptophan 741 were frequently identified in AIPC patients (Jeanny et al., 2007). There are a few available drugs, such as bicalutamide, enzalutamide, cabazitaxel, abiraterone acetate, and so on, used in the treatment of PCa, but still, newly developed incipient candidates were needed with high activities and lower drawbacks (Elancheran et al., 2016). The Food and Drug Administration (FDA) has recently approved the potent second-line agents, abiraterone, and enzalutamide. Abiraterone is a CYP17A1 inhibitor (blocking both 17α hydroxylase and 17,20-lyase, two enzymes important for androgen synthesis), while enzalutamide is a potent AR ligand binding domain (LBD) competitive antagonist that blocks nuclear translocation and AR-dependent gene transcription (Charles et al., 2018; Moses et al., 2018) and demonstrated efficacy against metastatic castrated resistance prostate cancer (CRPC) and late-stage clinical trials with advanced PCa (Jung et al., 2010; Scher et al., 2010). Apalutamide-509 is used for a high therapeutic index and has a protective effect for the treatment of PCa (Clegg et al., 2012; Rathkopf et al., 2013). Sipuleucel-T is the only immunotherapy currently available to prevent prostate cancer (Sims, 2012; Wesley et al., 2012). The structural modification and important interactions derived from the groups of flutamide (i), bicalutamide (ii), enzalutamide (iii), *N-(4-(4-hydroxyphenoxy)-3-methylphenyl)benzamide* (iv), and the designed molecule *(****6a-k****)* were shown in Figure 1.

**Figure 1:** Androgen receptor targeting therapeutics for the treatment of PCa.

Several studies are ongoing for the development of specific target-based drugs to minimize drug resistance, toxicity, dosage, and more (Veeramanikandan and Benita Sherine, 2015). *In vitro* anticancer activity of the synthesized hydrazide derivatives was determined against human colorectal (HCT116) cancer cells line. Recently, hydrazide derivative was reported as a potent and selective inhibitor for antibacterial–antifungal (Somashekhar, 2013; Popiołek, 2017), anti-inflammatory (Todeschini et al., 1998), antimalarial (Melnyk et al., 2006), and anti-tuberculosis activities (Bedia et al., 2006), as an Entamoeba histolyica (Afreen et al., 2016), a cruzipain inhibitor (Cerecetto and Gonzalez, 2010) and as Epidermal growth factor receptor (EGFR) Kinase Inhibitor (Wang et al., 2016). Thus, benzohydrazides are important moieties that exhibit more effective inhibitory activity against various cancer cell lines such as A549, MCF-7, HeLa, and HepG2 (Wang et al., 2016). The current study on benzohydrazide reveals it as an effective inhibitor for prostate cancer and its physicochemical properties. Some newly synthesized substituted fused pyrazolo, triazolo, and thiazolo pyrimidine derivatives were shown potent anti-prostate cancer activities with low toxicity comparable to bicalutamide as a reference drug (Bahashwan et al., 2014; Elancheran et al., 2017; Ferroni et al., 2017). The structure-based drug design approach for analyzing the structure-activity relationships (SAR) of molecules followed SAR studies (Antonella et al., 2013), which provided rules for the selection of new, potentially active compounds (Shvets and Dimoglo, 1999), which can be synthesized. In this study, we have reported the design and development of benzohydrazide derivatives as novel AR antagonists. The two combined substructures of the R-dihydronaphthalene-2-carbaldehyde ring and benzohydrazides might show synergistic anticancer effects. All these facts encouraged us to integrate these two moieties and screen new benzohydrazide derivatives as potential anti-prostate cancer agents. The compounds *(****6a-k****)* were synthesized and characterized by IR, NMR, and Mass Spectral techniques. Further, ***6g, 6j*, **and ***6k*** molecule structures were confirmed by single crystal XRD. The *in vitro* anticancer activities of the compounds *(****6a-k****)* were tested against LNCaP and PC3 cell lines (Divakar et al., 2017). The above remarkable considerations and pharmaceutical and industrial applications prompted us to synthesize a new series of benzohydrazide derivatives via the Schiff base route.

## Materials and Methods

### *In silico* Molecular Docking

The protein structure of AR (3V49) was obtained from Protein Data Bank (PDB) with the resolution of 1.70 Å bound with the ligand *4-[(4R)-4-(4-hydroxyphenyl)-3,4-dimethyl-2,5-dioxoimidazolidin-1-yl]-2-(trifluoromethyl)benzonitrile*, and prepared using Protein Preparation Wizard in Maestro 11.2. OPLS-2005 was used for the optimization and minimization until the root mean square deviation reached 0.3 Å. Then, Grid was generated using Grid generation Wizard for docking studies. The ligands were drawn and imported 2D structures to the Maestro project table. The 3D structures were prepared, geometrically refined, energy minimized, and assigned appropriate protonation state at pH 7.0 ± 2.0 using LigPrep module. The docking was carried out using GLIDE XP (extra precision method) (Maestro, 2016).

### Chemistry

All the reagents and solvents were obtained from commercial sources like Spectrochem, Merck, Alfa Aesar, Sigma-Aldrich, and used without further purification. The reactions were monitored by Merck silica gel 60 F254 thin layer chromatography (TLC) and visualized in a UV light chamber. Column chromatography was performed on Merck silica gel (100–200 mesh). Melting points were recorded by the open capillary method using Raagaa melting point apparatus. The FT-IR spectra using KBr pellets was recorded on a Thermo Scientific FT-IR spectrophotometer. In FT-IR spectra, the compounds exhibited the absorption bands at 3,250–3,150 cm^−1^ due to the presence of a secondary amine (NH) stretching, at 1,670–1,630 cm^−1^ due to amide (C = O) stretching, and at 1,605–1,590 cm^−1^ due to imine (C = N) stretching, which confirmed the formation of the compounds *(****6a-k****)*. Also, we found C-Cl stretching around 750–700 cm^−1^ and nitro stretching around 1,550 and 1,350 cm^−1^. The ^1^H and ^13^C NMR spectra were recorded by Bruker AVANCE II at 400 and 100 MHz, respectively using DMSO *d6* solvent at room temperature. In ^1^H NMR spectra, the compounds showed the amide proton signal at δ 11.9–12.3 ppm, CH = N- signal at δ 8.7–8.9 ppm, aromatic proton signals at δ 7.2–8.0 ppm, and 2 aliphatic CH_2_ protons signals at δ 2.5–3.0 ppm. In ^13^C NMR spectra, carbonyl (NH-C = O) signal was observed at δ 160–165 ppm, aromatic and CH = N- signals at 120–150 ppm, and aliphatic carbon signals at 20–30 ppm. Mass spectra were recorded using a JEOL GCMATE II LC-Mass spectrometer. The compounds showed significant parent ion peaks. High Performance Liquid Chromatography (HPLC) was used to identify the purity of the compounds, **6g** and **6j** as shown in Figures S3, S4. The melting point and yield of the compounds were illustrated in Table S1.

#### General Procedure for the Preparation of Benzoic Acid Hydrazide (*3a-3k*)

The substituted benzoic acid (0.01 mol) was taken in ethanol (10 ml) which had 2–3 drops of Conc. Sulfuric acid added to it. The reaction mixture was refluxed in 80°C for 7 h and monitored by TLC. After the completion, the reaction mixture was neutralized using sodium bicarbonate solution then extracted with ethyl acetate. The organic layer was evaporated and dried well. The product was purified by column chromatography using Ethyl acetate /Hexane as an eluent. To this, ester (2) was added with hydrazine hydrate (0.02 mol) in the presence of ethanol and refluxed in 80°C for 6 h. The completion of the reaction was monitored by TLC. Then, ethanol was removed, and ice-cold water was added. The white color precipitate was formed. Further, the precipitate was filtered and recrystallized from a suitable solvent (**3a-3k**).

#### Preparation of 1-chloro-3,4-dihydronaphthalene-2-carbaldehyde (5)

To the solution of 4-dihydronaphthalen-1(2H)-one (0.174 mol), the dry DMF and POCl_3_ (0.171 mol) was slowly added at 0°C and stirred for 30 min. The mixture was heated to 80°C for 2 h and transferred into the beaker containing 25% cold sodium acetate, then extracted with ether. The organic layer was evaporated and dried well to get residual oil, which solidified on cooling.

#### General procedure for the Preparation of Compounds (*6a-k*)

Benzohydrazide (0.01 mol) and 1-chloro-3,4-dihydronaphthalene-2-carbaldehyde (0.01 mol) were taken in ethanol (5 ml) with a few drops of acetic acid, refluxed for 8 h, then cooled to room temperature. The excess ethanol was removed through a high vacuum, and the residue was quenched with ice. The precipitate was filtered, dried, and further purified by column chromatography using ethyl acetate and hexane as eluent.

#### Experimental Data

The synthesized compounds *(****6a-k****)* were well-characterized by IR, NMR, and HRMS, and all the data are in accordance with the proposed structures as described below.

##### (E)-N'-((1-chloro-3,4-dihydronaphthalen-2-yl)methylene)benzohydrazide (6a)

Yield: 90%; mp: 168–170°C, pale white solid. FT-IR (KBr) ν max: 3204 (NH), 2938, 2851 (aromatic C-H), 1638 (amide C = O), 1592 (imine C = N) cm^−1^. ^1^H NMR (DMSO d_6_, 400 MHz, ppm): δ 12.10 (s, 1H, NH), 8.77 (s, 1H), 7.87 (d, *J* = 7.2, 2H), 7.64–7.25 (m, 7H), 2.808–2.764 (m, 4H). ^13^C NMR (DMSO d_6_, 100 MHz, ppm): δ 163.34, 143.77, 144.5, 136.97, 132.72, 132.63, 131.65, 130.73, 129.80, 129.49, 128.16, 128.00, 127.41, 124.94, 29.50, 26.54, 23.65, 21.51. Mass: *m/z* Calcd for C_18_H_15_ClN_2_O [M+H]^+^: 310.08; Found: 310.9758.

##### (E)-2-chloro-N'-((1-chloro-3,4-dihydronaphthalen-2-y**l**)methylene)benzohydrazide (6b)

Yield: 88%; mp: 168–170°C, pale white solid. FT-IR (KBr) ν max: 3184 (NH), 2940, 2894 (aromatic C-H), 1652 (amide C = O), 1594 (imine C = N) cm^−1^. ^1^H NMR (DMSO d_6_, 400 MHz, ppm): δ 12.9 (s, NH), 12.16 (s, NH), 8.70 (s, 1H, CH = N), 8.48 (s, 1H, CH = N), 7.34–7.72 (m, 16H, Ar H), 2.84–2.94 (m, 4H, (CH_2_)_2_), 2.74 (t, *J* = 4.8 Hz, 2H, CH_2_), 2.371 (t, *J* = 8 Hz, H2, 2H CH_2_). ^13^C NMR (DMSO d_6_, 100 MHz, ppm): δ 168.1, 159.5, 159.2, 158.8, 158.5, 157.3, 148.8, 133.9, 128.8, 127.9, 125.6, 121.2, 118.2, 115.2, 108.2, 58.9. Mass: *m/z* Calcd for C_18_H_14_Cl_2_N_2_O [M+H]^+^: 344.05; Found: 344.9302.

##### (E)-N'-((1-chloro-3,4-dihydronaphthalen-2-yl)methylene)-4-nitrobenzohydrazide (6c)

Yield: 85%; mp: 242–245°C; Green solid; FT-IR (KBr) ν max: 3165 (NH), 2918, 2849 (aromatic C-H), 1667 (amide C = O), 1601 (imine C = N) cm^−1^. ^1^H NMR (DMSO d_6_, 400 MHz, ppm): δ 12.39 (s, 1H), 8.845 (s, 1H), 8.39 (d, *J* = 8.8 Hz, 2H), 8.1735 (d, *J* = 8.4 Hz, 2H), 7.681–7.659 (m, 2H), 7.367–7.321 (m, 2H), 2.885–2.814 (m, 4H); ^13^C NMR (DMSO d_6_, 100 MHz, ppm): δ 161.86, 149.82, 147.9, 139.29, 138.10, 133.58, 132.52, 131.59, 129.7, 128.06, 127.47, 125.09, 29.49, 26.90, 23.61. Mass: *m/z* Calcd for C_18_H_14_ClN_3_O_3_ [M+H]^+^: 355.07; Found: 354.0069.

##### (E)-N'-((1-chloro-3,4-dihydronaphthalen-2-yl)methylene)-3-nitrobenzohydrazide (6d)

Yield: 86%; mp: 213–215°C; pale yellow solid. FT-IR (KBr) ν max: 3166 (NH), 2954, 2853 (aromatic C-H), 1669 (amide C = O), 1591 (imine C = N), 1536, 1348 (NO_2_) cm^−1^. ^1^H NMR (DMSO *d*_6_, 400 MHz, ppm): δ 12.333 (s, 1H), 8.843 (s, 1H), 8.783 (s, 1H), 8.469–8.446 (m, 1H), 8.4205 (d, *J* = 8 Hz, 1H), 7.875–7.835 (m, 1H) 7.676–7.653 (m, 2H), 7.360–7.315 (m, 2H), 2.882–2.815 (m, 4H); ^13^C NMR (DMSO *d*_6_, 100 MHz, ppm): δ 161.34, 148.27, 146.95, 138.05, 134.99, 134.67, 135.51, 132.53, 131.59, 130.82, 130.00, 128.04, 127.45, 126.90, 125.07, 122.77, 26.90, 23.62. Mass: *m/z* Calcd for C_18_H_14_ClN_3_O_3_ [M+H]^+^: 355.07; Found: 354.0234.

##### (E)-3-chloro-N'-((1-chloro-3,4-dihydronaphthalen-2-yl)methylene)benzohydrazide (6e)

Yield: 90%; mp: 208–210°C; pale pink solid. FT-IR (KBr) ν max: 3189 (NH), 2950, 2887 (aromatic C-H), 1648 (amide C = O), 1597 (imine C = N) cm^−1^. ^1^H NMR (DMSO *d*_6_, 400 MHz, ppm): δ 12.079 (s, 1H), 8.820 (s, 1H), 7.984 (s, 1H), 7.8965 (d, *J* = 7.6 Hz, 1H), 7.689–7.651 (m, 2H), 7.5885 (d, *J* = 7.6 Hz, 1H) 7.353–7.307 (m, 3H), 2.873–2.807 (m, 4H); ^13^C NMR (DMSO *d*_6_, 100 MHz, ppm): δ 162.03, 146.59, 138.59, 135.59, 133.79, 133.23, 132.55, 132.22, 131.65, 131.03, 129.94, 128.02, 127.79, 127.44, 127.03, 125.03, 26.91, 23.62. Mass: *m/z* Calcd for C_18_H_14_Cl_2_N_2_O [M+H]^+^: 344.05; Found: 344.9384.

##### (E)-N'-((1-chloro-3,4-dihydronaphthalen-2-yl)methylene)-4-methylbenzohydrazide (6f)

Yield: 92%; mp: 128–130°C; pale brown solid. FTIR (KBr) ν max: 3209 (NH), 2933, 2852 (aromatic C-H), 1635 (amide C = O), 1593 (imine C = N) cm^−1^. ^1^H NMR (DMSO *d*_6_, 400 MHz, ppm): δ 11.945 (s, 1H), 8.828 (s, 1H), 7.849 (d, *J* = 7.2, 2H), 7.663–7.642 (m, 1H), 7.344–7.296 (m, 5H), 2.831 (m, 4H), 2.088 (s, 3H); ^13^C NMR (DMSO *d*_6_, 100 MHz, ppm): δ 161.34, 145.77, 142.3, 137.97, 132.72, 132.63, 131.85, 130.73, 129.80, 129.49, 128.16, 128.00, 127.41, 124.96, 29.50, 26.94, 23.63, 21.51. Mass: *m/z* Calcd for C_19_H_17_ClN_2_O [M+H]^+^: 324.10; Found: 324.9966.

##### (E)-N'-((1-chloro-3,4-dihydronaphthalen-2-yl)methylene)-4methoxybenzohydrazide (6g)

Yield: 86%; mp: 190–192°C, Appearance—Cream solid. FTIR (KBr) ν max: 3222 (NH), 2952, 2840 (aromatic C-H), 1639 (amide C = O), 1605 (imine C = N) cm^−1^. ^1^H NMR (DMSO *d*_6_, 400 MHz, ppm): δ 11.928 (s, 1H), 8.812 (s, 1H), 7.9345 (d, *J* = 8.4, 2H), 7.657–7.636 (m, 1H), 7.340–7.295 (m, 3H), 7.068 (d, *J* = 8.8, 2H), 3.840 (s, 3H), 2.852–2.814 (m, 4H); ^13^C NMR (DMSO *d*_6_, 100 MHz, ppm): δ 162.31, 162.62, 145.41, 137.94, 132.65, 132.51, 131.89, 130.10, 129.75, 127.98, 127.45, 125.64, 124.91, 114.21, 55.9, 26.95, 23.67. Mass: *m/z* Calcd for C_19_H_17_ClN_2_O_2_ [M+H]^+^: 340.10; Found: 340.9898.

##### (E)-4-bromo-N'-((1-chloro-3,4-dihydronaphthalen-2-yl)methylene)benzohydrazide (6h)

Yield: 84%; mp: 238–240°C, Appearance—Light yellow solid. FTIR (KBr) ν max: 3215 (NH), 2955, 2842 (aromatic C-H), 1642 (amide C = O), 1595 (imine C = N) cm^−1^. ^1^H NMR (DMSO *d*_6_, 400 MHz, ppm): δ 12.098 (s, 1H), 8.814 (s, 1H), 7.8895 (d, *J* = 8.4, 2H), 7.7565 (d, *J* = 8.4, 2H), 7.6455 (d, *J* = 4.4 1H), 7.3105 (d, *J* = 10.8, 3H). 2.857–2.801 (m, 4H); ^13^C NMR (DMSO *d*_6_, 100 MHz, ppm): δ 162.59, 146.39, 136.01, 133.16, 132.68, 132.57, 132.02, 131.69, 131.22, 130.24, 129.89, 129.69, 128.01, 127.42, 126.22, 125.01, 26.33, 23.63. Mass: *m/z* Calcd for C_18_H_14_BrClN_2_O [M+H]^+^: 388.00; Found: 388.9875.

##### (E)-4-chloro-N'-((1-chloro-3,4-dihydronaphthalen-2-yl)methylene)benzohydrazide (6i)

Yield: 85%; mp: 238–240°C, Appearance—Light yellow solid. FTIR (KBr) ν max: 3210 (NH), 2945, 2849 (aromatic C-H), 1648 (amide C = O), 1592 (imine C = N) cm^−1^. ^1^H NMR (DMSO *d*_6_, 400 MHz, ppm): δ 12.086 (s, 1H), 8.801–8.790 (m, 1H), 7.944 (s, 2H), 7.6045 (d, *J* = 5.2, 3H), 7.310–7.270 (m, 3H), 2.805 (d, 4H); ^13^C NMR (DMSO *d*_6_, 100 MHz, ppm): δ 162.45, 146.36, 137.98, 137.24, 133.14, 132.55, 132.29, 131.66, 130.05, 129.87, 129.06, 128.25, 127.99, 127.39, 124.99, 26.90, 23.61. Mass: *m/z* Calcd for C_18_H_14_Cl_2_N_2_O [M-H]^+^: 344.05; Found: 343.0401.

##### (E)-N'-((1-chloro-3,4-dihydronaphthalen-2-yl)methylene)-4-hydroxybenzohydrazide (6j)

Yield: 86%; mp: 233–235°C, Appearance—Light yellow solid. FTIR (KBr) ν max: 3220 (NH), 2946, 2842 (aromatic C-H), 1652 (amide C = O), 1598 (imine C = N) cm^−1^. ^1^H NMR (DMSO *d*_6_, 400 MHz, ppm): δ 11.857 (s, 1H), 10.216 (s, 2H), 8.795 (s, 1H), 7.834 (d, 2H), 7.650–7.628 (m, 1H) 7.330–7.269 (m, 3H), 6.8775 (d, *J* = 8.4, 2H), 4.428–4.403 (m, 1H), 2.847–2.85 (m, 4H); ^13^C NMR (DMSO *d*_6_, 100 MHz, ppm): δ 163.18, 161.31, 145.17, 137.91, 132.67, 132.37, 131.92, 130.25, 129.70, 127.96, 127.38, 124.89, 124.08, 115.52, 26.96, 23.68. Mass: *m/z* Calcd for C_18_H_15_ClN_2_O_2_ [M-H]^+^: 326.08; Found: 325.0741.

##### (E)-3-bromo-N'-((1-chloro-3,4-dihydronaphthalen-2-yl)methylene)benzohydrazide (6k)

Yield: 86%; mp: 218–220°C, Appearance—Pale Yellow. FTIR (KBr) ν max: 3220 (NH), 2946, 2842 (aromatic C-H), 1652 (amide C = O), 1598 (imine C = N) cm^−1^. 1H NMR (DMSO, 400 MHz, ppm): δ 2.860–2.793 (m, 4H), 12.099 (s, 1H), 8.805 (s, 1H), 7.343–7.284 (m, 3H), 7.526–7.486 (m, 1H), 7.660–7.638 (m, 1H), 8.115 (s, 1H), 7.9411–7.922 (m, 1H), 7.826–7.796(m, 1H). ^13^C NMR (DMSO, 100 MHz, ppm): δ 161.97, 146.58, 138.02, 135.77, 135.10, 133.27, 132.55, 131.64, 131.26, 130.62, 129.32, 128.01, 127.42, 125.03, 122.24, 26.91, 23.62, 21.22. Mass: *m/z* Cal.cd for C_18_H_15_ClN_2_O [M+H]^+^: 388.00; Found: 388.9874.

### Single Crystal X-Ray Diffraction Studies

The single crystal X-ray diffraction data of ***6g, 6j*, **and ***6k*** was recorded at the University of Mysore, India (Bruker axs kappa apex2, CCD diffractometer using graphite monochromated MoK radiation). The structure was solved by SHELXS-97 and refined by full-matrix least square methods in SHELXL-97. All non-hydrogen atoms were refined anisotropically and the hydrogen atoms were refined isotropically.

### Biological Evaluation

#### Anti-proliferation Assay

The *in vitro* antiproliferation activities were performed by using prostate cancer cell lines (LNCaP & PC-3) obtained from the National Center for Cell Science (NCCS), Pune, India. The cells were cultured in RPMI medium with 10% FBS and incubated at 37°C with 5% CO_2_. Approximately 5,000 cells/well were seeded into a 96 well cell culture plate. The antiproliferation activities of the compounds were tested by adding different concentrations and incubated for 48 h to evaluate the activities. Then, 10 μL of MTT (5 mg/ml) was added to each well and incubated for an additional 4 h, and the absorbance was measured at 560 nm. The experiments were performed in triplicates, and the standard deviation was calculated (Hayon et al., 2003; Chen, 2011).

#### Acridine Orange (AO)/Ethidium bromide (EtBr) Dual Staining for Apoptosis

For conventional AO/EtBr apoptosis assay 5X10^5^ cells/well were seeded in a 6 well plate and incubated at 37°C and 5% CO_2_ for overnight. The cell lines were treated with the test compound for 48 h. The concentration of dye was prepared as a 1:1 ratio. Each dye concentration was 100 μg/ml. Cells were stained with 8 μL of dye for 5 min, and images were taken immediately by fluorescence microscopy (Maliheh et al., 2012; Tayyaba et al., 2016).

#### Western Blot

The LNCaP cells were cultured in medium supplemented with 10% charcoal-stripped FBS. The cells were treated for 24 h with ARA3 (1 μM) or bicalutamide (10 μM) in the presence or absence of 1 nM DHT. The cells were lysed by RIPA buffer supplemented with protease and phosphatase inhibitor cocktail. The lysate was centrifuged at 16,000 g for 20 min. The supernatant equivalent to 40 μg of protein was subjected to SDS PAGE gel electrophoresis. The resolved proteins were transferred to a PVDF membrane. The transferred proteins were then hybridized with antibodies, AR (sc816) or p-AR213 (sc135635) or procaspase-3 (sc7148) or akt1 (sc5289) or p-akt1 473 (sc293125) antibodies. The expression of β-actin was measured as an internal control using β-actin antibody (ab8227). The proteins were detected by horseradish peroxidase-labeled anti-rabbit or anti-mouse IgG monoclonal or polyclonal antibody, and a chemiluminescence detection kit (ECL, GE healthcare). The intensities of the PCR product in the agarose gel 402 were scanned with G: BOX (Syngene) image scanner.

#### DNA Methyl Transferase Enzyme Inhibitor (DNMT) Assay

A DNMT inhibition assay was carried out using EpiQuik DNA methyltransferase activity/inhibition screening assay kit (Epigentek, Brooklyn, NY, USA) according to the manufacturer's instruction. Two different concentrations of each test compound were screened using the Enzyme-linked immunosorbent assay (ELISA) kit. Their enzyme inhibitory activity was quantified by colorimetric assay method. The assay was performed in duplicates for each concentration (Robertson, 2002).

### Pharmacokinetic Properties Prediction (ADME)

The two-dimensional structures of the compounds *(****6a-k****)* were imported to the Maestro project table and minimized using LigPrep. The program, Qikprop40 module (Schrödinger software) was used for the *in silico* determination of pharmacokinetic properties. A preliminary test of the drug-likeness of the compounds was calculated in accordance with Lipinski's rule of five. To obey Lipinski's rule of five and rule of three, the compounds required molecular weight (mol_MW) of less than 500 amu, not more than 5 and 10 hydrogen bond donors (Donor HB), hydrogen bond acceptors (Accpt HB), the partition coefficient between octanol and water (QPlogPo/w) to be <5, (QPlogS > −5.7), (QPPCaco > 22 nm/s) and, respectively, primary metabolities < -5.7. The compounds which have more than one violation of these rules are not considered as orally active molecules. The properties such as IC_50_ value for the blockage of HERG K+ channels, the percentage of human oral absorption, blood-brain barrier permeability, and aqueous solubility were also predicted to identify the bioactivity of the compounds.

### Molecular Dynamics

Molecular Dynamic (MD) stimulation studies were carried out by Desmond (2012) module of Schrödinger software. The docked conformer of benzohydrazides with a good Glide-score was chosen for the Molecular Dynamics simulations study with an OPLS-2005 force field. The protein-ligand complex was bounded with a predefined TIP3P water model (Jorgensen et al., 1983) in orthorhombic box. The volume of the box was minimized, and the overall charge of the system was neutralized by adding Na^+^ and Cl^−^ ions. The pressure and temperature were kept constant at 300 K and 1.01325 bar using Nose-Hoover thermostat (Hoover, 1985) and Martyna-Tobias-Klein barostat (Martyna et al., 1994) methods. The simulations were performed using NPT ensemble by considering number of atoms, pressure, and timescale. During simulations, the long-range electrostatic interactions were calculated using the Particle-Mesh-Ewald method (Essmann et al., 1995). The Root Mean Square Deviation (RMSD) was used to measure the average change in displacement of a selection of atoms for a particular frame concerning a reference frame. This was calculated for all structures in the trajectory.

## Results and Discussion

### Molecular Docking

A molecular docking approach was followed for designing of benzohydrazide derivatives by using Schrödinger (Maestro 11.2) software (Maestro, 2016). The 3D structure of the human androgen receptor alpha ligand binding domain with the Selective Androgen Receptor Modulators (SARM) inhibitor *(PDB ID: 3V49)* was obtained from the Protein Data Bank, refined the structure and was used for the study (Nique et al., 2012; Lakshmithendral et al., 2019). Docking studies were carried out to find the potential binding affinity and the interaction between the compounds ***(6a-k***) and AR protein, as shown in Figure S1. Compounds (6a-k) have van der Waals interactions with surrounding hydrophobic residues TRP741, LEU873, ARG752, MET747, MET749, VAL746, MET745, LEU873, MET742, PHE876, VAL903, ILE899, ILE898, LEU701, LEU704, LEU707, PHE891, and form hydrogen bonds through a hydrazide group with two residues LEU704, HIE 876 in the Helix 12. The highest scoring pose of compound ***6j*** and the drug bicalutamide from docking studies is shown in Figure 2 with receptor residues. From docking studies, we found that the compound ***6j*** showed the highest glide score (−11.776 kcal/mol) and glide energy of −52.02 kcal/mol, respectively. Compounds *(****6a-k****)* also showed binding affinity to AR, and their docking scores are shown in Table 1. The compounds *(****6b, 6d, 6a, 6g****)* also have higher binding energy in the range of −10.767 to −9.893 kcal/mol and glide energy vary from −49.591 to −44.96 kcal/mol. The standard Bicalutamide glide score was −11.064 kcal/mol and binding energy was −44.712 kcal/mol, respectively. These studies were conventional, and the results were reported.

**Figure 2:** Predicted binding mode of compound **6j (A,C)** and standard Bicalutamide **(B,D)** in AR LBD (PDB: 3V49) highlighting the H-bond, Pi-Pi stacking, and specific hydrophobic interactions.

**Table 1:** Predicted binding energy and mode of the compounds, ***6a-k***.

**Compounds**	**Glide gscore**	**Glide evdw**	**Glide ecoul**	**Glide energy**	**Interacting residues**
6a	−10.407	−43.292	−1.668	−44.96	TRP741, PHE764
6b	−10.767	−45.192	−2.009	−47.201	–
6c	−8.521	−46.952	−0.51	−47.462	PHE764
6d	−10.701	−40.531	−2.456	−41.987	LEU704, PHE764, TRP741
6e	−7.682	−47.995	−0.766	−48.761	–
6f	−7.41	−46.602	−0.732	−47.334	TRP741
6g	−9.893	−47.783	−1.528	−49.311	–
6h	−7.434	−49.335	−0.256	−49.591	–
6i	−10.572	−45.596	−1.691	−47.287	PHE764, TRP741
**6j**	**−11.776**	**−46.559**	**−5.46**	**−52.02**	**HIE874**, **TRP741**
6k	−9.925	−32.985	−0.146	−33.131	TRP741
Bicalutamide	−11.064	−42.986	−1.726	−44.712	ARG752, TRP741

*Glide evdw, van der Waals interaction energies; Glide ecoul, Coulomb interaction energies. Bold values indicate the highest docking score*.

### Chemistry

Molecular docking scores intend the synthesis of the compounds *(****6a-k****)*. The series of compounds were synthesized, as shown in Scheme 1. The substituted benzoic acid was first converted to their corresponding ester (esterification) followed by refluxing with hydrazine hydrate in ethanol at 80°C for 6–7 h, which resulted in the formation of acid hydrazides *(****3a-k****)* (Chidananda et al., 2012). 1-chloro-3,4-dihydronaphthalene-2-carbaldehyde (5) was prepared by using alpha-tetralone (4) under 0–5°C with reagents DMF and POCl_3_ (Perumal et al., 2012). Further, the compounds *(****6a-k****)* were obtained by the reaction of compounds *(****3a-k****)* with 1-chloro-3,4-dihydronaphthalene-2-carbaldehyde (5) refluxing in the presence of ethanol for 14–16 h (Rapartia et al., 2009; Sirisoma et al., 2009). All the compounds were purified by column chromatography, and their structures were confirmed with spectral techniques. The melting point and yield of the compounds were shown in Table S1. The compounds, ***6g, 6j*, **and ***6k*, **were crystallized by slow evaporation at room temperature in DMSO/chloroform, ethanol/acetonitrile solvents (Sheldrick, 1997). The compound ***6g*** belongs to the monoclinic system with space group belonging to *P2*_1_*/a*, a = 8.431(3) Å, b = 15.653(5) Å, c = 12.771(4) Å, α = 90°, β = 97.522(12)°, γ = 90°, Z = 4. The compound ***6j*** belongs to the monoclinic system with space group belonging to *P*2_1_/*c*, a = a = 5.2090 (4) Å, b = 25.128 (2) Å, c = 12.7739 (10) Å, α = 90°, β = 96.138(2)°, γ = 90°, Z = 2. Similarly, the compound ***6k*** belongs to a Tetragonal system with space grouping I 41/*a*, a = 22.136 (3) Å, b = 22.136 (5) Å, c = 14.5289 (4) Å, α = 90°, β = 90°, γ = 90°, Z = 16 (Sheldrick, 1990, 2015). The ORTEP diagram of the compounds ***6g, 6j*, **and ***6k*** were illustrated in Figure 3. The unit cell diagram of the compounds ***6g, 6j*, **and ***6k*** are shown in Figure S2. The details of the crystal data and structure refinement parameters were summarized in Tables S2–S4. The purity of compounds ***6g*** and ***6j*** were analyzed using HPLC. The compound ***6g*** showed the purity of 99.42%, and ***6j*** had the purity of 99.90% as illustrated in Figures S3, S4. All the spectroscopic measurements confirm the compounds' structures and purity.

**Scheme 1:** Synthesis of benzohydrazide derivatives.

**Figure 3:** ORTEP structure of Compounds **6g**, **6j**, and **6k**.

### Biological Evaluation

The compounds *(****6a-k****)* were evaluated for the anticancer activities against the prostate cancer cell lines (PC-3, LNCaP) and non-cancerous cell line (3T3), as compared with the standard, Bicalutamide by using MTT assay (Divakar et al., 2017). The results demonstrated that the compounds *(****6a-k****)* showed significant cytotoxic potential in PC-3 and LNCaP cell lines in the IC_50_ range of 7–38 μM, as compared with Bicalutamide (IC_50_-11.06), listed in Table 2. Of these compounds, the ***6g*** and ***6j*** exhibited significant dose-dependent activities in LNCaP cell lines (IC_50_ 7.17 ± 1.87 and 10.45 ± 0.7, respectively) and PC-3 (IC_50_ 32.09 ± 0.86 and 44.65 ± 0.32, respectively). The percentage of cell viability of the compound, ***6g*** in LNCaP and PC-3 cell lines were shown in Tables S5, S6. The anticancer activities were shown in Figures S5, S6 by plotting percentage cell viability against the concentration of the compounds. These studies suggests that the methoxy group at R influenced the anticancer activities (Plouvier et al., 1995). In addition, the replacement of the hydroxyl group at R slightly decreased the IC_50_ value. Similarly, the nitro group at R showed less IC_50_ value, when compared with the hydroxyl group. The compounds, ***6g*** and ***6j*** did not show the toxicity against 3T3 cells line, which reliably represents normal human mammary cells. From the series, ***6g*** and ***6j*** showed more promise for anti-prostate cancer activity in LNCaP and PC-3 cell lines. It is evident that the groups, especially OCH_3_, OH, and NO_2_ substitutions, showed more anticancer activities in the cell proliferation assays. The compound ***6g*** exhibited dose-dependent activity in LNCaP cell lines. Analysis of the AO/EtBr staining revealed that the synthetic compound ***6g*** reduced cell viability of LNCaP cell lines and induced the apoptosis. Chromatin condensation and Cell membrane blebbing is the first phase of cell disassembly during apoptosis, which was observed in the treatment group. Live cells had normal nuclei staining, which presented green chromatin with organized structures. Apoptotic cells containing condensed or fragmented chromatin (green or orange) are shown in Figure 4. As described earlier, the western blotting analysis was carried out and is shown in Figure S7. The androgen significantly increased the protein expression of AR (~1.2 fold) and p-AR 213 (~1.4 fold), compared to the control (Saravanan et al., 2017). Bicalutamide and ***6g*** significantly decreased the androgen-stimulated AR and p-AR protein expression. The notable difference between bicalutamide and ***6g*** is that ***6g*** could significantly decrease the protein expression of p-AKT (~0.7 fold) and procaspase-3 (~0.6 fold), while bicalutamide treatment did not show a significant effect on those proteins. The significance (*P* < 0.05) was obtained by applying one-way Analysis of Variance (ANOVA) followed by a *post-hoc* turkey test, as shown in Figure 5. The compound ***6g*** showed DNMT1 enzyme inhibitory activity at 1 and 100 μM concentration, as shown in Table 3. A concentration gradient response was observed, and the high concentration exhibited 23.9% in the enzyme inhibition assay. So, this compound can be used for DNMT1 isoform targeted therapies to treat prostate cancer.

**Table 2:** Bioactivity of test and standard compounds.

**Ligand**	LNCaP (μM)^*^, ^a^ (T877A AR)	**PC3 (μM)^a^(AR–)**	**3T3 (μM)^a^ (non-cancer)**	**SelectivityAR–/AR+**	**Safety 3T3/LNCaP**
6a	>100	>100	>100	–	–
6b	21.68 ± 4.84	40.41 ± 3.88	48.17 ± 2.03	1.86	2.22
6c	12.34 ± 1.38	43.20 ± 1.65	>100	–	–
6d	14.16 ± 0.64	48.20 ± 2.87	54.21 ± 1.68	3.40	3.8
6e	18.56 ± 1.49	48.56 ±1.73	50.21 ± 1.63	2.61	2.7
6f	>100	>100	>100	–	–
**6g**	**7.17** **±** **1.87**	**32.09** **±** **0.86**	>100	–	–
6h	>100	>100	>100	–	–
6i	21.56 ± 1.37	43.94 ± 1.82	50.87 ± 2.55	2.03	2.35
6j	**10.45** **±** **0.7**	**44.65** **±** **0.32**	>100	–	–
6k	38.57 ± 1.29	72.14 ± 1.25	>100	–	–
Bicalutamide^b^	26.3 ± 0.07	58.26 ± 1.86	62.55 ± 0.32	2.21	2.37

* *IC_50_ of the compounds stimulated by 1nM DHT*.

a *The values are the mean ± standard deviation (SD) of three independent experiments performed in triplicate*.

b *Positive control*.

*Bold values indicate the highly active compound*.

**Figure 4:** The morphological changes in **6g** and Zebularine treated in prostate cancer cell line. The treated and untreated cells were stained with Acridine orange and Ethidium bromide and observed under an inverted fluorescent microscope. Live cells appear green, late apoptotic cells are appearing orange in color, and necrotic cells are colored red.

**Figure 5:** **AR**: DHT significantly (#) increased the AR expression compared to control. Bicalutamide and **6g** significantly (^*^) reduced the DHT stimulated expression of AR. **p-AR**: DHT significantly (##) increased the p-AR 213 expression compared to control. Bicalutamide and **6g** significantly (^*^) reduced the DHT stimulated expression of p-AR 213. **AKT:** Expression of AKT1 protein. There is no significant difference with the treatments. **p-AKT: 6g** significantly (^*^) reduced the DHT stimulated expression of p-AKT1 473. **Procaspase-3: 6g** significantly decreases the expression of procaspase-3 compared to control. The experiments were conducted in duplicates and the average value was represented as mean ± S.D. The significance (*P* < 0.05) was obtained by applying one way ANOVA followed by *post-hoc* turkey test. (^***^P < 0.001, ^**^P < 0.01, ^*^ *P* < 0.05).

**Table 3:** DNMT inhibition assay.

**DNMT 1 Inhibition assay**				
**Test compound**	**1** **μM**		**100** **μM**	
	**OD** **±** **SD**	**% Inhibition**	**OD** **±** **SD**	**% Inhibition**
Control	1.519 ± 0.062			
5AZA	1.329 ± 0.022	12.5	0.922 ± 0.096	39.3
6g	1.318 ± 0.810	13.2	1.157 ± 0.446	23.9

### ADME

Several drugs are failed during clinical trials due to poor adsorption, distribution, metabolism, and elimination properties, so ADME was paid large attention in drug discovery. It was utilized for the screening and optimization of active compounds *(****6a-k****)*. The ADME has an important role in the assessment of drug-likeness and pharmacokinetic properties. We have analyzed all the predicted ADME parameters, such as hydrogen bond acceptors (Acceptor HB), hydrogen bond donors (Donor HB), molecular mass, and so on, as shown in Table S7. All the compounds fell under Lipinski's rule of five and pharmacokinetic properties. There were no more than 5 hydrogen bonds donors, 10 hydrogen bond acceptors, and all molecules masses had <500 Daltons. All the compounds had a good percentage of human oral absorption. The IC_50_ value of HERG K+ (channel blockage (−6.2 to −6.9), (QPlogHERG) of all the tested compounds showed a good range of values (Schrödinger., 2019 -1). In this study, the compounds obeyed the recommended drug-likeness properties and were orally active. All the pharmacokinetics results were in good agreement with previous reports.

### Molecular Dynamic Simulations

The benzohydrazide-3V49 complex was immersed in the orthorhombic box with a TIP3P water solvent model used for simulations using OPLS-2005 force field. After the solvent system was formed, the simulation was equilibrated for 5 ns by Dynamic simulation (Anand et al., 2015). The quality study of the simulations was performed as depicted in Table 4. The root mean square deviation (RMSD) plots are shown in Figure 6 indicating the benzohydrazide−3V49 complex reached its stable form. Protein RMSD started from 0.8 Å and later stabilized at 1.4 Å, whereas, in ligand RMSD started from 2.4 Å and stabilized around 1.5 Å. Changes of the order of 1–3 Å are perfectly acceptable for small, globular proteins. Changes much larger than that, however, indicate that the protein is undergoing a large conformational change during the simulation. It is also important that simulation converges; the RMSD values stabilize around a fixed value. The nitrogen atom of the hydrazide ring displayed hydrogen bond interaction with LEU704 (68%) and ASN705 (20%), and bridged with H_2_O. The current geometric criteria for the protein-ligand H-bond is: a distance of 2.5 Å between the donor and acceptor atoms (D—H•••A); a donor angle of 120° between the donor-hydrogen-acceptor atoms (D—H•••A); and an acceptor angle of 90° between the hydrogen-acceptor-bonded atoms (H•••A—X). The π-π stacking interaction was also observed with TRP 741 (74%) and PHE764 (73%) in the binding pocket of 3V49. The 2D interaction poses, and the histogram chart are depicted in Figure 7.

**Table 4:** Summary of simulation quality analysis after equilibration.

**S. no**.	**Properties**	**Statistical parameters**
1	Simulation period [ns]	5.008
2	Degrees of freedom	35123
3	Number of atoms	28514
4	Average total energy [kcal/mol]	45199.046
5	Average potential energy [kcal/mol]	55518.371
6	Temperature [K]	300
7	Pressure [bar]	14.244
8	Volume [Å^3^]	56247.958

**Figure 6:** The RMSD plot obtained for compound ***6g*** *and* ***3V49*** complex.

**Figure 7:** The histogram chart and the percentage of interactions in molecular dynamic simulations.

## Conclusion

In this present study, a series of molecules were designed by the molecular docking approach for androgen receptors. The binding affinities of the ligand and the precise interactions, molecular dynamics simulations validate the results of molecular docking. Further, the compounds *(****6a-k****)* were synthesized and demonstrated anti-prostate cancer activity. The compounds ***6g*** and ***6j*** were the most promising among the series, especially against LNCaP cell lines, IC_50_ values 7.17 ± 1.87 and 10.45 ± 0.7 μM, respectively. Also, the compounds ***6a-j*** were screened against 3T3 cells line for the toxicity. The binding energy of compounds ***6g*** and ***6j*** with the androgen receptor were significantly noticeable (−49.311 and −52.02 kcal/mol). Moreover, it is evident from the results that the methoxy and hydroxy substitutions at R have better binding affinities and anticancer activities than others. Also, the compound ***6g*** significantly decreased the mRNA expression of AR-stimulated genes and induced apoptosis. We intend to further investigate the target site and study the *in vivo* anticancer activity of the active compounds.

## Data Availability

All datasets generated for this study are included in the manuscript and/or the Supplementary Files.

## Author Contributions

HA, RE, and SK conceived and designed the experiment. HA and NM performed the experiment. HA, RE, and KL analyzed the data. HA and RE wrote the manuscript. MR and AB have done a critical revision of the manuscript for important intellectual content. NL carried out the analysis of single crystal XRD structures. All authors have contributed to the final version and approved the final manuscript.

### Conflict of Interest Statement

The authors declare that the research was conducted in the absence of any commercial or financial relationships that could be construed as a potential conflict of interest.

## Supplementary Material

Supplementary data associated LCMS and NMR spectra of compounds, *(****6a-k****)*. The Crystallographic data for compound ***6g, 6j*, ***and* ***6k*** have been deposited with the Cambridge Crystallographic Data Center, **CCDC No. 1878869, 1916916**, and **1903192**. Copies of the data can be obtained free of charge on application to CCDC, 12 Union Road, Cambridge CB2 1EZ, UK (fax: 044 (0) 1223 336033 or deposit@ccdc.cam.ac.uk).
